The article "Quantum Decoherence Technique for Two Two-level Interacting Atomic Engineering in Dissipative Field" was published in 2022. Journal: Comput Intell Neurosci.

# Quantum Decoherence Technique for Two Two-level Interacting Atomic Engineering in Dissipative Field

**DOI:** 10.1155/2022/7987716

**Published:** 2022-05-29

**Authors:** Pengli Shu

**Affiliations:** Department of Physics, Lvliang University, Lvliang, Shanxi 033000, China

## Abstract

In order to improve the in-depth understanding and research on the dissipative field of atomic engineering, the research object of this paper is the dissipative field of atomic engineering. Through the engineering of two two-level interacting atoms as the background, an in-depth study of two two-level atoms is carried out, so the decoherence factor of two two-level atoms is obtained. In this paper, the numerical simulation calculation experiment of the dissipative field of atomic engineering is carried out, and the evolution of the quantum coherent oscillation of the dissipative field to the quantum decoherence is discussed. The results indicate that the dissipation coefficient and strength of the atom-light field interaction not only affect the oscillation of the quantum coherent evolution of atomic states but also the periodicity of the evolution. All preliminary results throw light on the nature of two-level interacting atoms in the dissipative field of atomic engineering, which also provides a reference value for related researchers.

## 1. Introduction

With the continuous social and economic development, the studies on quantum mechanics have become more and more in-depth gradually [1–5]. Quantum entanglement is a unique property of quantum mechanics and its essential application in the field of quantum information science, which has attracted the increasing attention of humans [6–8]. On the one hand, atoms can be used to store and process quantum information and photons can be used to transmit quantum information. However, nonlinear interaction is the physical foundation for quantum entanglement. Hence, the interaction between the light field and atoms is considered to be stored in the ideal carrier for processing quantum information [9–11]. The interaction between two atoms induced by the nonresonant interaction of the two atoms and the cavity field can be used to implement the Grover search. However, under the large detuning conditions, when the single-mode optical cavity has energy address loss, with respect to the evolution features of entropy in the single-mode radiation field and the interaction system of two two-level atoms, the impact of the cavity field loss on the dynamic is significant. Hence, it is of great significance to study the impact of the cavity field loss on the dynamic behavior of the light field interacting with two two-level atoms [12, 13].

The article "Quantum Decoherence Technique for Two Two-level Interacting Atomic Engineering in Dissipative Field" was published in 2022. Journal: Comput Intell Neurosci.

In recent years, as the term quantum has gradually moved from behind the scenes to the front, the practical application of quantum mechanics has also appeared in all aspects of human life. Quantum decoherence refers to the process in which a coherent quantum state becomes an incoherent quantum state under the influence of the outside world (such as environmental noise). It includes properties such as open quantum systems, quantum entanglement of quantum and environment, and loss of coherence over time. In this paper, the quantum decoherence technology in the dissipation field of two two-level interacting atoms engineering is analyzed based on the quantum theory. Through digital analysis and calculation, the impact of the coupling intensity coefficient *g* and the dissipation constant between the cavity field and the atom on the evolution of the quantum coherence in the atomic state is discussed [14–17].

## 2. Model and Solution

The system is radiation field. After the light field is quantized, from the perspective of the basic principle of the interaction between light and atoms, the general Hamiltonian of field interaction of the atom and light in the case of nonresonant interaction can be obtained. When it is far away from resonance, that is, in a large detuning situation ($\Delta =\omega -\omega_{0}\gg g\sqrt{n}$, in which Δ stands for the amount of atom-field detuning, *ω* stands for the frequency of the light field, after the rotation wave is approximated and subject to adiabatic eliminated. The effective Hamiltonian can be obtained as (*η* = 1):

(1) $$\begin{array}{c} H=\lambda \left[\sum_{j=1,2}\left({|1\rangle }_{j},\langle 1|aa^{+}-{|0\rangle }_{j},\langle 0|a^{+}a\right)+\left(S_{1}^{+}S_{2}^{-}+S_{1}^{-}S_{2}^{+}\right)\right]. \end{array}$$

In the above equation, *λ*=*g*^2^/Δ, in which *a*+*a* stands for the generation (annihilation) operator of the light field, and *S*_*j*_(*j*=1,2) stands for the artificial spin operator of the j-th atom.

### 2.1. The Characteristics of the Loss Field

If the cavity field loss is considered, the density operator of the system shall meet the master equation as the following:

(2) $$\begin{array}{c} \frac{\text{d}\rho \left(t\right)}{\text{d}t}=-i\left[H,\rho \left(t\right)\right]+D\rho \left(t\right). \end{array}$$

In the above equation, *Dρ*(*t*) describes the energy loss of the cavity field, which can be written as the following:

(3) $$\begin{array}{c} D\rho \left(t\right)=k\left[2a\rho \left(t\right)a^{+}-a^{+}a\rho \left(t\right)-\rho \left(t\right)a^{+}a\right]. \end{array}$$

In the above equation, *k* is the decay coefficient.

It is assumed that at the initial moment, the light field is in a coherent state as the following:

(4) $$\begin{array}{c} |\varphi_{F}\left(0\right)\rangle =\left|\alpha \rangle \;=e^{-\left(1/2\right){\left|\alpha \right|}^{2}}\sum_{n=0}^{\infty }\frac{\alpha^{n}}{\sqrt{n!}}n\rangle \;\right|. \end{array}$$

The atoms are in an entangled state as the following:

(5) $$\begin{array}{c} \left|\varphi_{A}\left(0\right)\rangle \;=\sin\;\theta \right|\left|{0\rangle \;}_{1}{0\rangle \;}_{2}+\cos\;\theta \right|{1\rangle \;}_{2}. \end{array}$$

In the above equation, |0〉 and |1〉 stand of a single atom, respectively. The density operator of the system at the initial moment is as the following:

(6) $$\begin{array}{c} \rho_{F,A}\left(0\right)=\;\sin^{2}\theta \left|00,\alpha \rangle \;\langle \;\alpha ,00||+|\sin|\theta |\;|\cos|\theta |\left|00,\alpha \rangle \;\langle \;\alpha ,00\right||+|\;|\cos^{2}|\theta ||\mathrm{\alpha ,}11\rangle \;\langle \;11\text{,}\alpha \right|. \end{array}$$

Under the initial conditions given by equation (6), in an interaction scene, through equation (2), the density can be obtained as the following:

(7) $$\begin{array}{c} \rho_{F,A}\left(t\right)=\alpha_{1}\left|00,\alpha \left(t\right)e^{-2i\lambda t}\rangle \;\langle \;\alpha \left(t\right)e^{-2i\lambda t}\alpha ,00||+|a_{2}||00,\alpha \left(t\right)e^{-2i\lambda t}\rangle \;\langle \;\alpha \left(t\right)e^{-2i\lambda t}\alpha ,11\right|+a_{3}\left|11,\alpha \left(t\right)e^{-2i\lambda t}\rangle \;\langle \;\alpha \left(t\right)e^{-2i\lambda t}\alpha ,00||+|a_{4}||11,\alpha \left(t\right)e^{-2i\lambda t}\rangle \;\langle \;\alpha \left(t\right)e^{-2i\lambda t}\alpha ,11\right|. \end{array}$$

The reduced density operator of the atom at time *t* can be obtained by tracing the light field as the following:

(8) $$\begin{array}{c} \rho_{A}\left(t\right)=tr_{F}\left(\rho \left(t\right)\right)=a_{1}\left|00\rangle \;\langle \;00||+|a_{2}|\exp|\left[-{\left|\alpha \left(t\right)\right|}^{2}\left(1-e^{-4i\lambda t}\right)\right]||00\rangle \;\langle \;11\right|+a_{3}\exp\left[-{\left|\alpha \left(t\right)\right|}^{2}\left(1-e^{4i\lambda t}\right)\right]\left|11\rangle \;\langle \;00||+|a_{4}||11\rangle \;\langle \;11\right|. \end{array}$$

In general, the coherence phenomenon indicates that the nondiagonal element is not zero. However, the modulus of the nondiagonal element is of practical significance. Hence, from equation (8), it is not difficult to obtain the decoherence factor as the following:

(9) $$\begin{array}{c} f\left(\lambda ,\alpha ,k,t\right)=\left|e^{-2i\lambda t}\exp\left[\frac{k}{k+2i\lambda }\left(1-e^{-2\left(k+2i\lambda \right)t}\right){\left|\alpha \right|}^{2}\right]\times \;\exp\left[-{\left|\alpha \right|}^{2}\left(1-e^{-2ikt}\right)\right]\times \;\exp\left[-{\left|\alpha \left(t\right)\right|}^{2}\right]\left(1-e^{-4i\lambda t}\right)\right|. \end{array}$$

After simplification, the following can be obtained:

(10) $$\begin{array}{c} f\left(\lambda ,\alpha ,k,t\right)=\exp\left[\frac{k{\left|\alpha \right|}^{2}}{k^{2}+4\lambda^{2}}\cdot \left[k+e^{-2kt}\left(2\lambda \;\sin\;4\;\lambda t-k\;\cos\;4\;\lambda t\right)\right]\right]\times \;\exp\left[-{\left|\alpha \right|}^{2}\left(1-e^{-2kt}\right)\right]\times \;\exp\left[-{\left|\alpha \right|}^{2}e^{-2kt}\left(1-\cos\;4\;\lambda t\right)\right]. \end{array}$$

From equation (10), the reduced density operator of the atom can be obtained as the following

(11) $$\begin{array}{c} \rho_{a}\left(t\right)=Tr_{f}\rho \left(t\right)=C_{11}\left|1,1|\rangle \;|\langle 1,1||+|C_{22}|\exp|\left[-{\left|\alpha \left(t\right)\right|}^{2}\left(1-e^{-2i\Omega t}\right)\right]||1,1\rangle |\langle \;|1,0\right|+\\ C_{13}\exp\left[-{\left|\alpha \left(t\right)\right|}^{2}\left(1-e^{-2i\Omega t}\right)\right]\left|1,1|\rangle \;|\langle 0,1||+|C_{14}|\exp|\left[-{\left|\alpha \left(t\right)\right|}^{2}\left(1-e^{-4i\Omega t}\right)\right]||1,1\rangle |\langle \;|0,0\right|+\\ C_{21}\exp\left[-{\left|\alpha \left(t\right)\right|}^{2}\left(1-e^{2i\Omega t}\right)\right]\left|1,0|\rangle \;|\langle 1,1||+|C_{22}||1,0\rangle |\langle 1,0||+|C_{23}||1,0\rangle |\langle \;|0,1\right|\\ C_{24}\exp\left[-{\left|\alpha \left(t\right)\right|}^{2}\left(1-e^{-2i\Omega t}\right)\right]\left|1,0|\rangle \;|\langle 0,0||+|C_{31}|\exp|\left[-{\left|\alpha \left(t\right)\right|}^{2}\left(1-e^{2i\Omega t}\right)\right]||0,1\rangle |\langle \;|1,1\right|+\\ C_{32}\left|0,1|\rangle \;|\langle 1,0||+|C_{33}||0,1\rangle |\langle 0,1||+|C_{34}|\exp|\left[-{\left|\alpha \left(t\right)\right|}^{2}\left(1-e^{2i\Omega t}\right)\right]||0,1\rangle |\langle \;|0,0\right|+\\ C_{41}\exp\left[-{\left|\alpha \left(t\right)\right|}^{2}\left(1-e^{4i\Omega t}\right)\right]\left|0,0|\rangle \;|\langle 1,1||+|C_{42}|\exp|\left[-{\left|\alpha \left(t\right)\right|}^{2}\left(1-e^{-2i\Omega t}\right)\right]||0,0\rangle |\langle \;|1,0\right|+\\ C_{43}\exp\left[-{\left|\alpha \left(t\right)\right|}^{2}\left(1-e^{2i\Omega t}\right)\right]\left|0,0|\rangle \;|\langle 0,1||+|C_{44}||0,0\rangle |\langle \;|0,0\right|. \end{array}$$

From equation (10), the reduced density operator of the light field can be obtained as the following

(12) $$\begin{array}{c} \rho_{f}\left(t\right)=T_{\tau_{\alpha }}\rho \left(t\right)=C_{11}\left|\alpha \left(t\right)e^{-2i\Omega t}|\rangle \;|\langle \;|\alpha \left(t\right)e^{-2i\Omega t}\right|+C_{22}\left|\alpha \left(t\right)|\rangle \;|\langle \alpha \left(t\right)||+|C_{33}||\alpha \left(t\right)\rangle |\langle \alpha \left(t\right)||+|C_{44}||\alpha \left(t\right)e^{2i\Omega t}\rangle |\langle \;|\alpha \left(t\right)e^{2i\Omega t}\right|. \end{array}$$

From equation (10), the system can be obtained as the following

(13) $$\begin{array}{c} S\left(t\right)=1-T_{T}\rho^{2}\left(t\right)=\frac{1}{2}\left(\sin^{2}\theta_{1}+\;\sin^{2}\theta_{2}\right)-\frac{3}{8}\sin^{2}\theta_{1}\sin^{2}\theta_{2}-\frac{1}{2}\left(\sin^{2}\theta_{1}+\;\sin^{2}\theta_{2}-\;\sin^{2}\theta_{1}\sin^{2}\theta_{2}\right)\times \\ \exp\left\{\left[\frac{2k^{2}}{k^{2}+\Omega^{2}}\left(1-e^{-2kt}\cos\;2\;\Omega t\right)+\frac{2k\Omega }{k^{2}+\Omega^{2}}e^{-2kt}\text{sin}2\Omega t\right]{\left|\alpha \right|}^{2}\right\}\exp\left[-2{\left|\alpha \right|}^{2}\left(1-e^{-2kt}\right)\right]-\\ \frac{1}{8}{\text{sin}}^{2}\theta_{1}{\text{sin}}^{2}\theta_{2}\text{exp}\left\{\left[\frac{2k^{2}}{k^{2}+4\Omega^{2}}\left(1-e^{-2kt}\cos\;4\;\Omega t\right)+\frac{4k\Omega }{k^{2}+4\Omega^{2}}e^{-2kt}\sin\;4\;\Omega t\right]{\left|\alpha \right|}^{2}\right\}\\ \times \text{exp}\left[-2{\left|\alpha \right|}^{2}\left(1-e^{-2kt}\right)\right]. \end{array}$$

From equation (12), the linear entropy of the light field can be obtained as the following

(14) $$\begin{array}{c} S_{f}\left(t\right)=1-Tr_{f}\rho_{f}^{2}\left(t\right)=\frac{1}{2}\left(\sin^{2}\theta_{1}+\;\sin^{2}\theta_{2}\right)-\frac{3}{8}\sin^{2}\theta_{1}\sin^{2}\theta_{2}\\ -\frac{1}{2}\left(\sin^{2}\theta_{1}+\;\sin^{2}\theta_{2}-\;\sin^{2}\theta_{1}\sin^{2}\theta_{2}\right)\times \\ \exp\left[-2{\left|\alpha \right|}^{2}e^{-2kt}\left(1-\cos\;2\;\Omega t\right)\right]-\frac{1}{8}\sin^{2}\theta_{1}\sin^{2}\theta_{2}\exp\left[-2{\left|\alpha \right|}^{2}e^{-2kt}\left(1-\cos\;4\;\Omega t\right)\right]. \end{array}$$

Taking into consideration a system consisting of two entangled ideal cavities (C1 and C2) and two independent two-level Rydberg atoms (A1 and A2), atom A1 passes through one cavity C1, and atom A2 passes through the other cavity C2, as shown in Figure 1 below. Based on the theory of the J-C model, the field composite system under the rotating wave approximation is shown as the following:

(15) $$\begin{array}{c} H_{J}=g\left(a_{1}\sigma_{+}^{\left(1\right)}+a_{1}^{+}\sigma_{-}^{\left(1\right)}+a_{2}\sigma_{+}^{\left(2\right)}+a_{2}^{+}\sigma_{-}^{\left(2\right)}\right). \end{array}$$

In the above equation, *g* stands for the interaction coupling intensity coefficient of the atomic cavity field; *a*+ and a stand of each cavity field; *σ*^+^(*σ*^−^) stand for the spin operators of each atom. Without considering the atom dissipation, if only the cavity field dissipation is taken into account, the dynamic evolution equation of the composite system in the interaction painting can be obtained based on equation (16) as the following:

(16) $$\begin{array}{c} \dot{\rho }=\dot{\rho }{\left|{}_{\text{atorn}-\text{field}}+\dot{\rho }\right|}_{\text{field}-\text{reservoir}}. \end{array}$$

In which,

(17) $$\begin{array}{c} {\dot{\rho }}_{\text{atom}-\text{feild}}=-i\left[H_{1},\rho \right]\\ =-ig\left(a_{1}\sigma_{+}^{\left(1\right)}\rho +a_{1}^{+}\sigma_{-}^{\left(1\right)}\rho -\rho a_{1}\sigma_{+}^{\left(1\right)}-\rho a_{1}^{+}\sigma_{-}^{\left(1\right)}+a_{2}\sigma_{+}^{\left(2\right)}\rho +a_{2}^{+}\sigma_{-}^{\left(2\right)}\rho -\rho a_{2}\sigma_{+}^{\left(2\right)}-\rho a_{2}^{+}\sigma_{-}^{\left(2\right)}\right)\\ {\dot{\rho }|}_{\text{field}-\text{reservoir}}=-k_{1}\left(a_{1}^{+}a_{1}\rho -2a_{1}\rho a_{1}^{+}+\rho a_{1}^{+}a_{1}\right)-k_{2}\left(a_{2}^{+}a_{2}\rho -2a_{2}\rho a_{2}^{+}+\rho a_{2}^{+}a_{2}\right). \end{array}$$

In the above equation, k1 and k2 stand for the dissipation coefficients of the cavities C1 and C2, respectively. It is assumed that the eigenstates of the two single-mode cavity fields have only |0〉 and |1〉, and they are initially ${|\psi \left(t=0\right)\rangle }_{c_{1}c_{2}}=\left(1/\sqrt{2}\right)\left(|0_{1}1_{2}\rangle +|1_{0}0_{2}\rangle \right)$. The two atoms are initially in the respective ground states |*ψ*(*t*=0)〉_*A*_1__=|*g*_1_〉 and |*ψ*(*t*=0)〉_*A*_2__=|*g*_2_〉. In addition, the atom and the cavity field fall into the coherent resonance interaction. The initial state wave function of the aforesaid composite system is shown as the following:

(18) $$\begin{array}{c} \left|{\psi \left(t=0\right)\rangle \;}_{C_{1}C_{2}A_{1}A_{2}}=\frac{1}{\sqrt{2}}\left(\left|0_{1}1_{2}\rangle \;\langle \;1_{1}0_{2}\right|\right)⊗\right|g_{1}g_{2}\rangle \;, \end{array}$$

where the high-order terms of k/g are ignored, the density operator of the system can be solved based on equations (15)–(18) as the following:

(19) $$\begin{array}{c} \rho {\left(t\right)}_{C_{1}C_{2}A_{1}A_{2}}=\alpha_{1}\left|0_{1}1_{2}g_{1}g_{2}|\rangle \;|\langle 0_{1}1_{2}g_{1}g_{2}||+|\alpha_{2}||0_{1}1_{2}g_{1}g_{2}\rangle |\langle \;|0_{1}1_{2}g_{1}g_{2}\right|\\ +\alpha_{3}\left|1_{1}0_{2}g_{1}g_{2}|\rangle \;|\langle 1_{1}0_{2}g_{1}g_{2}||+|\alpha_{4}||0_{1}1_{2}g_{1}g_{2}\rangle |\langle \;|0_{1}1_{2}g_{1}g_{2}\right|+\\ \alpha_{5}\left|0_{1}1_{2}g_{1}g_{2}|\rangle \;|\langle 1_{1}0_{2}g_{1}g_{2}||+|\alpha_{5}||1_{1}0_{2}g_{1}g_{2}\rangle |\langle \;|0_{1}1_{2}g_{1}g_{2}\right|+\\ \alpha_{6}\left|0_{1}1_{2}g_{1}g_{2}|\rangle \;|\langle 0_{1}1_{2}g_{1}g_{2}||+|\alpha_{6}||0_{1}1_{2}g_{1}g_{2}\rangle |\langle \;|0_{1}1_{2}g_{1}g_{2}\right|. \end{array}$$

Based on equation (19), the reduced density matrix of the two atoms can be obtained as the following:

(20) $$\begin{array}{c} \rho {\left(t\right)}_{A_{1}A_{2}}=Tr_{C_{1}C_{2}}\rho \left(t\right)=\left(\alpha_{1}+\alpha_{3}\right)\left|g_{1}g_{2}|\rangle \;|\langle g_{1}g_{2}||+|\alpha_{2}||g_{1}e_{2}\rangle |\langle \;|g_{1}e_{2}\right|\\ +\alpha_{4}\left|e_{1}g_{2}|\rangle \;|\langle e_{1}g_{2}||+|\alpha_{6}||g_{1}e_{2}\rangle |\langle g_{1}e_{2}||+|\alpha_{6}||e_{1}g_{2}\rangle |\langle \;|g_{1}e_{2}\right|. \end{array}$$

With the engineering of two two-level interacting atoms as the background, the quantum decoherence in the resonance interaction process of two two-level atoms with two entangled single-photons in the dissipative cavity field is studied to obtain the decoherence factor of two two-level atoms. Through the numerical simulation calculation, the evolution of the quantum coherence oscillation of the dissipation field to quantum decoherence is explored.

The article "Quantum Decoherence Technique for Two Two-level Interacting Atomic Engineering in Dissipative Field" was published in 2022. Journal: Comput Intell Neurosci.

## 3. Simulation Calculation and Discussion

When the two atoms are in the ground state (*θ*_1_=*θ*_2_=*π*) or the excited state (*θ*_1_=*θ*_2_=0) at the initial moment, the linear entropy of the atom-light field system, the atom, and the light field is always zero. The reason is that in the case of large detuning.

The position of fluid particles is evenly distributed, and the velocity is randomly distributed according to the system temperature. The state of solid wall particles is given according to the specific boundary conditions. The macro flow parameters are obtained by statistical method, and the sampling time length is related to the equilibrium process. In this paper, 104 time steps are taken, the flow area is 20 × 20, 800 fluid particles, and 120 solid particles are arranged, which is recommended according to the literature. The DPD particle number density is between 2 and 10, which is taken as 2 in this paper. The horizontal motion velocities V of the upper plate are 012, 118, and 5, respectively.

From equations (13)–(15), it can be known that the linear entropy of the atom-light field system, the atom, and the light field are all related, and the evolution of each linear entropy corresponding to various initial states of the atoms is also different with the extension of time. When the two atoms are in the ground state (*θ*_1_=*θ*_2_=*π*) or the excited state (*θ*_1_=*θ*_2_=0) at the initial moment, the linear entropy of the atom-light field system, the atom, and the light field is always zero. The reason is that in the case of large detuning, it can be known from equations (10) to (12) that when *θ*_1_=*θ*_2_=*π*, *ρ*_*f*_(*t*)=|*α*(*t*)*e*^2*i*Ω*t*^〉 〈 *α*(*t*)*e*^2*i*Ω*t*^|, *ρ*_*α*_(*t*)=|0,0〉 〈 0,0|, *ρ*(*t*)=*ρ*_*α*_(*t*) ⊗ *ρ*_*f*_(*t*). From the above equations, the light field is at |*α*(*t*)*e*^±2*i*Ω*t*^〉, and its amplitude decays exponentially.

The article "Quantum Decoherence Technique for Two Two-level Interacting Atomic Engineering in Dissipative Field" was published in 2022. Journal: Comput Intell Neurosci.

At the initial moment, if *θ*_1_=0 and *θ*_2_=*π*, the following can be obtained based on (10)

(21) $$\begin{array}{c} \rho \left(t\right)=\frac{1}{2}\left[\left(1+\cos\;2\;\Omega t\right)|1,0,\alpha \left(t\right)\rangle \langle 1,0,\alpha \left(t\right)|+i\;\sin\;2\;\Omega t|1,0,\alpha \left(t\right)\rangle \langle 0,1,\alpha \left(t\right)|\right.\\ \left.-i\;\sin\;2\;\Omega t|0,1,\alpha \left(t\right)\rangle \langle 1,0,\alpha \left(t\right)|+\left(1-\cos\;2\;\Omega t\right)|0,1,\alpha \left(t\right)\rangle \langle 0,1,\alpha \left(t\right)|\right]=\\ \left\{\left(\cos\;\Omega t|1,0\rangle -i\;\sin\;\Omega t|0,1\rangle \right)\left(\cos\;\Omega t\langle 1,0|+i\;\sin\;\Omega t\langle 0,1|\right)\right\}⊗|\alpha \left(t\right)\rangle \langle \alpha \left(t\right)|. \end{array}$$

If Ω*t*=*π*/4 is selected, the following can be obtained:

(22) $$\begin{array}{c} \rho \left(t\right)=\frac{1}{2}\left\{\left.\left(\left|1,0|\rangle \;|-|i||0,1\rangle \right)\left(\langle 1,0|+i\langle \;0,1|\right.\right)\right\}|⊗|\left\{|\alpha \left(t\right)\rangle \langle \alpha \left(t\right)|\right\}|=||\psi_{EPR}\rangle |\langle \psi_{EPR}||⊗|\left\{|\alpha \left(t\right)\rangle \langle \;\alpha \left(t\right)|\right.\right\}. \end{array}$$

From the above analysis, it can be seen that under the aforesaid conditions, the prepared EPR pair does not decay in the whole evolution process. The reason is that the dipole interaction between atoms leads to entanglement between atoms (which can be observed from equation (1)), and there is always no photon exchange between the light field and the atomic system. Hence, the loss of the light field only results in the exponential decay of the amplitude of the light field but does not lead to the decay of the atomic EPR pair.

At the initial moment, the two atoms are in a state of equal probability superposition; that is, when the sum of the distribution angles *θ*_1_ and *θ*_2_ of the two atoms are both *π*/2, the linear evolution pattern of the atom-light field system, the atoms, and light fields over time can be obtained from equations (13) to (15). The linear entropy of the system is greater than zero at any time, except the initial time when it is zero, and it increases with the extension of time. When it increases to a certain level, it tends to stabilized to a specific value. The time from zero to a stable value is reduced with the increase of the decay constant. The magnitude of the stable value is related to the average photon number |*α*|^2^ of the light field and increases with the increase of |*α*|^2^; the linear entropy of the atom presents an oscillation situation with decreasing amplitude, and the oscillation stops after a period of time, which makes the linear entropy of the atom tend to be linear with the system at the stable value of the same entropy, and its oscillation time is quickly reduced with the increase of the decay constant. Due to the large detuning interaction between the atoms and the light field, the dynamic Stark shift and the atomic dipole-dipole interaction of the atomic system that is dependent on the light field occur in the atomic system. The shift of different atomic energy levels is not the same. As a result, the reduced density operator of the light field in the field interaction system evolves periodically between the pure state and the mixed state in atom-light interaction. Hence, the linear entropy of the light field shows periodic oscillation with decreasing amplitude, and the oscillation period is *π*/Ω. At *t*_*d*_=*nπ*/Ω(*n*=1,2, ⋯), *S*_*f*_(*t*_*d*_)=0, *S*_*a*_(*t*_*d*_)=*S*(*t*_*d*_) > 0, where the oscillation stops after a period of time. The linear entropy of the light field tends to reduce to zero; its oscillation time is related to the decay constant, reduced with the increase of the decay constant, and extended with the increase of the average photon number of the light field). From the above analysis, it can be seen that the system and atoms are in a mixed state at all times except at the initial moment when it is in a pure state, and the degree of mixing remains unchanged after a period of time. At the moment of *t*_*d*_, the light field is completely decoupled from the atom, and the light field is reduced to the original pure state. However, the atoms are still in a mixed state.

The article "Quantum Decoherence Technique for Two Two-level Interacting Atomic Engineering in Dissipative Field" was published in 2022. Journal: Comput Intell Neurosci.

The nondiagonal element of the density matrix can be used to describe the coherence of the quantum system, in which the nondiagonal element is not 0, suggesting that there is a coherence phenomenon. The decoherence factor can be expressed by the modulus of the nondiagonal element. Hence, the decoherence factor between two atoms can be obtained based on equation (22) as the following:

(23) $$\begin{array}{c} F\left(g,k,t\right)=\left|\frac{1}{2}\left(e^{-k_{1}t/2}\text{sin}gt-\frac{k_{1}e^{-k_{1}t/2}}{2g}+\frac{k_{1}}{2g}\right)\times \left(e^{-k_{2}t/2}\text{sin}gt-\frac{k_{2}e^{-k_{2}t/2}}{2g}+\frac{k_{2}}{2g}\right)\right|. \end{array}$$

From equation (23), it can be easily observed that the decoherence factor is related to the atom-light field coupling constant and the cavity field dissipation coefficient. In order to understand the evolution of the decoherence factor *f* (*g*, *k*, *t*) over time more clearly, a numerical analysis was performed (shown in Figures 2–6).

As shown in Figure 2, under the circumstance where the system does not have any dissipation (*k*1 = *k*2 = 0), the amplitude of the decoherence factor F remains unchanged with the extension of time, with a maximum value of 1 and a minimum value of 0. When the decoherence factor *F* = 1, the coherence is the most intense, and when *F* = 0, the coherence disappears. From Figures 3–6, the situation where there is dissipation in the cavity field can be observed (k/g≠0). From Figures 3–6, it can be seen that the decoherence factor presents the amplitude-reducing oscillation.

After a certain period of time, it becomes stabilized to the value 0, when the phenomenon of complete decoherence appears. The system evolves from the initial pure state to the final mixed state. In addition, it can be found that although the decoherence factor presents an overall amplitude decay situation, it does not keep decaying all the time, but the amplitude may increase occasionally. Moreover, it can also be observed that the larger the value of k/g is, the shorter the time for the amplitude it takes to decay to 0, which suggests that the influence of the dissipation coefficient in the light field on the coherence is apparent.

## 4. Conclusion

In this paper, the evolution features of quantum coherence between the atoms and single-photons in the resonant atomic states in two entangled ideal cavities and the time evolution features of the atomic-light field system linear entropy, the atomic linear entropy, and the light field linear entropy are studied. The impacts of the initial state of the two atoms, the decay constant, and the average photon number of the light field on each linearity are discussed. The results indicate that the dissipation factor and the intensity of the atom-light field interaction can affect not only the oscillation of the quantum coherence evolution in the atomic state but also the periodicity of the evolution. The decoherence factor presents an amplitude-reducing oscillation and tends to be stabilized at a value of 0 after a certain period of time, with the occurrence of a complete decoherence phenomenon.

## Figures and Tables

**Figure 1:** System where two atoms in the ground state pass through the C1 and C2 cavities in the maximum entangled state at the same time.

**Figure 2:** Diagram of the changes in the decoherence factor between two atoms with gt when *k*1 = *k*2 = 0.

**Figure 3:** Diagram of the changes in the decoherence factor between two atoms with gt when *k*1 = *k*2 = 0.05 g.

The article "Quantum Decoherence Technique for Two Two-level Interacting Atomic Engineering in Dissipative Field" was published in 2022. Journal: Comput Intell Neurosci.

**Figure 4:** Diagram of the changes in the decoherence factor between two atoms with gt when *k*1 = *k*2 = 0.1 g.

**Figure 5:** Diagram of the changes in the decoherence factor between two atoms with gt when *k*1 = 0.1 g, *k*2 = 0.05 g.

**Figure 6:** Diagram of the changes in the decoherence factor between two atoms with gt when *k*1 = 0.1 g, *k*2 = 0.2 g.

## Data Availability

The data used to support the findings of this study are available from the corresponding author upon request.
